RETRACTED

# Evaluation of periimplant bone neoformation using different scanning electron microscope methods for measuring BIC. A dog study

**DOI:** 10.4317/jced.50624

**Published:** 2012-02-01

**Authors:** José L. Calvo-Guirado, Antonio Aguilar-Salvatierra, Javier Guardia, Rafael Delgado-Ruiz, María P. Ramírez-Fernández, Cristina Pérez Sánchez, Gerardo Gómez-Moreno

**Affiliations:** 1 Department of Implant Dentistry, School of Medicine and Dentistry, University of Murcia, Spain; 2 Department of Pharmacological Interactions in Dentistry, Dental School, University of Granada, Spain; 3 Master of Implant Dentistry. Faculty of Medicine and Dentistry, University of Murcia

## Abstract

Objetives: The aim of this study was to determine which of three methods for measuring BIC (bone-to-implant contact), using vestibular and lingual scanning electron microscopy (SEM) for different implant systems at 15, 30 and 90 days post-surgery was the most precise. An elemental analysis with SEM was used to evaluate neoformed bone composition for three implant systems at the same study times. Material and Methods: 36 implants were placed in eighteen Beagle dogs mandible about one year old and weighing approximately 12-13 kg in order to evaluate bone apposition to three different implant surfaces. It was used the third and fourth premolar and ﬁrst molar distal sockets in both quadrants of the mandible (3P3, 4P4 and 1M1). Teeth were hemi-sected and the distal roots were removed. The specimens were prepared for histological examination and each section surface was stained using Masson’s trichrome and hematoxylin and eosin stains. BIC evaluations were performed by the three methods, BIC I (the quantity of mineralized bone in direct contact with the implant’s titanium surface across the entire threaded area); BIC II (along a line that passes from apex to apex of the implant threads); BIC III (both in areas around and above the threads and in between threads). Results: Both BIC and bone content were analyzed for all implants placed in P3, P4 y M1 alveoli on both, the buccal and palatine sides (elemental analysis quantified Ca, P, O and C). It was seen it was only at the ninety-day mark that high percentages of calcium were present. Conclusions: This study suggest that BIC III evaluation is the most certain method for establishing the quantity of bone formed as the BIC area.

** Key words:**Bone-to-impant contact, dogs, extraction socket, implants.

## Introduction

Most research in the field of implantology is concerned with evaluating bone-to-implant contact (BIC) as this is the chief factor contributing to implant stability. Numerous authors have specified the factors influencing BIC levels, in particular: original bone density, functional force values exerted on implants, implant materials and shape, surface roughness, implant length and width (1-5). But to date no study has responded to the question of what the best method for evaluating BIC might be, nor have any studies set out to assess the reliability of the various methods of evaluating BIC currently in use.

RETRACTED

It is a well-known fact calcium levels are a good indicator of bone quality, so elemental analysis is a good way of assessing the quality of neoformed bone (6-7). Although there may be good BIC levels, if the neoformed bone is of low quality with low calcium content, implant retention will be less than expected and long-term stability may be compromised (8). Studies involving elemental analysis used for this purpose are few; indeed, our review of studies involving BIC evaluation have identified only one that includes elemental analysis.

The aim of this study was, firstly, to determine which of three methods for measuring BIC using vestibular and lingual scanning electron microscopy (SEM) for different implant systems at fifteen, thirty and ninety days post-surgery was the most precise and, secondly, carry out elemental analysis using SEM to evaluate neoformed bone composition for the three implant systems at the same study times.

## Material and Methods

There are three different ways of measuring bone-to-implant contact. The first consists of measuring the quantity of mineralized bone in direct contact with the implant’s titanium surface across the entire threaded area. This we will call BIC I. It measures new bone around the implant threads but does not measure the new bone that joins this to old bone. BIC II measures BIC along a line that passes from apex to apex of the implant threads; this measures real BIC but does not take into account BIC between threads. This tends to measure old bone and some new bone but ignores inter-thread bone. Lastly, BIC III measures BIC both in areas around and above the threads and in between threads (Fig.1).

**Figure 1:** BIC measurement (a) BIC I, (b) BIC II, (c) BIC III.

This experimental animal study was designed in order to evaluate bone apposition to three different implant surfaces: a) 36 Certain Nanotite Implants 4 x 10 mm (Biomet 3i, Palm Beach Gardens, FL, USA), b) 36 SPI implants 3.5 x 9.5 mm (Thomen Medical, Waldenburg, Switzerland) c) 36 Evolution 2 implants 4 x 10 mm (B & W S.R.L, Buenos Aires, Argentina) placed in canine mandibles. The surfaces of the Certain implants were treated using the usual double acid etching with DCD; the SPI implant is a modified SLA implant with hydroxide ions to provide high surface energy and the Evolution 2 was also treated with double acid etching.

RETRACTED

Eighteen Beagle dogs about one year old and weighing approximately 12–13 kg each were used in the experiment. The animals were fed a daily pellet diet. The Ethics Committee for Animal Research at the University of Murcia, Spain, approved the three study protocols following guidelines laid down by the European Union Council Directive of November 24th, 1986 (86/609/EEC).

Surgical procedure

Implants were placed under the same surgical conditions as the tooth extractions in terms of sterility, operating theatre and anesthesia (Fig. 2). Six implants were placed into each mandible according to a random distribution pattern (www.randomization.com) established for each dog prior to surgery. The small sulcular ﬂaps were adapted for tension-free wound closure with interrupted and horizontal mattress sutures.

**Figure 2:** Inmediate Implant Placement.

During the ﬁrst week following surgery, the animals received Amoxicillin (500mg, twice daily) and Ibuproprofen 600mg (three times a day) via the systemic route. Sutures were removed after two weeks and dogs were submitted to oral hygiene during the process of osseointegration. The animals were sacriﬁced at two, four and twelve weeks after the implantation procedure by means of an overdose of Pentothal Natrium (Abbot Laboratories). The mandibles were dissected and each implant site was removed using a diamond saw (Exact Apparatebeau, Norderstedt, Hamburg, Germany). Biopsies were processed for ground sectioning according to the meth-ods described by Donath and Breuner (9). Histological and histomorphometric analyses were performed in order to evaluate bone quality and BIC on each side (vestibular and palatine).

Histologic Preparation, Histomorphometric Analysis and Histological Examination.

The most central sagittal section of each implant was used for histomorphometric analysis using MIP 4 software 4 (Microm Image Processing Software, CID, Consulting Image Digital, Barcelona, Spain) connected to a Sony color video camera DXC-151 2/3-CCD RGB. Each section surface was stained using Masson’s trichrome stain and hematoxylin and eosin stain (Fig. 3).

**Figure 3:** Histological sections to evaluate bone union: (a, d), B&W; (b, e), 3i and (c, f), Thomen medical.

Histomorphometric analysis was carried out using a scanning electron microscope (JEOL-6100- X LINK-ISIS, Akishima, Tokyo, Japan). Digital images were obtained with x100 magnification and processed with Imaris 6.1.5. software (Bitplane AG, Zurich, Switzerland) . Bone-to-implant contact was calculated for each sample using the three methods described earlier, BIC I, BIC II and BIC III.

Statiscical analysis

Elemental analysis values were taken from each of the central implant threads on the vestibular and lingual sides of each sample. Statistical analysis evaluated differences in elemental composition (Ca, P, O, C) between the three different BIC measurement methods (BIC I, BIC II and BIC III) were evaluated. Normality tests were applied: the Shapiro-Wilk test, the Student t-test or the Anova for two independent variables, as well as the Mann-Whitney and Wilcoxon (nonparametric) homogeneity of variance tests using SPSS 15.0 for Windows software (detection of significant differences and standard deviation), taking 5% as significant.

RETRACTED

## Results

Elemental analysis using BIC I at the fifteen-day mark found the greatest quantities of calcium and phosphorous in the lingual zone of P3. With BIC II, most calcium and phosphorous were found in the lingual zone of P3 whilst the greatest quantities of oxygen were found in the buccal zone of P3. However, when BIC III was analyzed it was found that calcium and phosphorous levels were greater at M1 than around the premolars.

At thirty days, with BIC I and BIC II, higher percentages of calcium and phosphorous were found in the buccal zones of P4 and the lingual area of M1. With BIC III, the highest percentages of calcium and phosphorous were found in the buccal zone of P3 and M1.

In the elemental study carried out at ninety days, with BIC I the highest percentages of calcium, phosphorous and oxygen were found in the buccal zone of P3. With BIC II, calcium, phosphorous and oxygen were greater at P3 than at P4 and M1. And with BIC III, the highest percentages of calcium, phosphorous and oxygen were buccal of P4. Carbon was found in higher quantities in the lingual zone of M1.

When the Mann-Whitney test was applied in order to compare calcium levels found with BIC I and BIC II, 119 samples were included, the average was 50.40 for BIC I and 69.44 for BIC II. For comparing phosphorous levels present there were 57 samples for BIC I and 55 for BIC II, the averages being 47.37 and 65.96 respectively. For oxygen, there were a total of 120 samples, averages being 59.50 for BIC I and 61.50 for BIC II. Finally, for carbon, the same number of samples were included for BIC I and BIC II (58 each) and the averages were 65.82 and 51.18 respectively. Mann-Whitney U test results were: 1203.5 for calcium, 1047 for phosphorous, 1740 for oxygen and 1257.5 for carbon. Wilcoxon W test results were: 2973.5 for calcium, 2700 for phosphorous, 3570 for oxygen and 2968.5 for carbon ( Table 1).

**Table 1:** Statistical test comparisons for BIC I and BIC II

When calcium data obtained from BIC I and BIC III readings was compared, including 59 and 49 samples re-spectively, the averages were 48.19 with BIC I and 62.10 with BIC III. For phosphorous there were a total of 106 samples, the averages being 47.98 with BIC I and 59.92 with BIC II. For oxygen there was a total of 120 samples with averages of 62.73 with BIC I and 58.28 with BIC III. Lastly, carbon levels were compared between 58 BIC I samples and 57 BIC III samples producing averages of 61.59 and 54.34 respectively. Mann-Whitney U test and Wilcoxon W test results can be observed in  Table 2.

RETRACTED

**Table 2:** Statistical test comparisons for BIC I y BIC III

Finally, comparing calcium content data between BIC II BIC III findings, there were 60 BIC II samples and 49 BIC III samples producing averages of 57.24 with BIC II and 52.26 with BIC III. For phosphorous, a total 104 samples were included and averages were 55.75 with BIC II and 48.66 with BIC III. For oxygen there were 120 samples (60 BIC II and 60 BIC III) and averages obtained were 63.23 with BIC II and 57.78 with BIC III. Lastly, for carbon there were 58 BIC II samples and 57 BIC III samples, averages being 54.17 and 61.89 respectively. Mann-Whitney U test and Wilcoxon W test results can be observed in  Table 3.

**Table 3:** Statistical test comparisons for BIC II and BIC III

## Discussion

Bone-to-implant contact is a sine qua non condition for the osteointegration of dental implants. It is a fact that bone-to-implant contact will not be the same in the palatine zone as in the buccal zone, as less contact is pro-duced on the buccal side this being a finer bone wall (10). Most of the research referenced in the present study only evaluate BIC in palatine areas, producing sets of values that are not altogether certain; generating averages based on this data alone assumes that BIC percentages will be the same all over the implant surface when this clearly not the case.

Very few studies describe how BIC has been measured. Roriz enter into details of how they evaluated BIC but point out that measurements were taken mesially and distally but we believe that collecting data from these sites cannot be completely significant as there will probably be similar amounts of bone on the mesial and distal sides (11).

Fenner evaluated BIC differentiating between buccal and lingual readings but measured BIC according to the height of the residual bone whilst in the present study we measured post-extraction BIC (12). They demonstrated that if residual bone height is of two millimeters then BIC will be greater on the buccal side but if it is of four, six or eight millimeters, BIC will be greater on the palatine side. Vignoletti, Song, Alexander and Parlar expressed BIC as an average of data taken on vestibular and lingual sides (13-16). We are in full agreement with this method as it does produce reliable data.

RETRACTED

Most research uses optical microscopes for taking histomorphometric evaluations but this is not an exact method for obtaining BIC values as measurement is taken from a photo of the microscope image. With the scanning electron microscope measurement can be carried out directly without the need for intermediary digital imagery. Only studies by Vidigal, Lee and Jeong take BIC measurements using SEM, whilst authors who have used light microscopes include: Calvo-Guirado, Orsini and Fenner (12,17-23).

With regard to elemental analysis, a single study by Ballo carries out elemental analysis of bone tissue in contact with the implant surface (24). Their analysis utilized BIC I evaluation and found that Calcium and Phosphorous were the principle elements present in this tissue. In the present study elemental composition was evaluated at three study periods (at fifteen days, thirty days and ninety days) for the three BIC evaluation approaches. At all study times carbon and oxygen were the predominant elements with small quantities of Calcium and Phosphorous.

## Conclusion

Calcium percentages evaluated by the three BIC evaluation methods and over the three study periods were found to differ widely. Elemental analysis was carried out on old bone in order to establish a pattern/model of normality, as a control, and it was seen it was only at the ninety-day mark that high percentages of calcium were present. In the rest of the samples, independently of the BIC evaluation method, calcium was found to be present in very small quantities, indicating that the neoformed bone was of poor quality, particularly with BIC I at ninety days.

It must be said that BIC III evaluation is the most certain method for establishing the quantity of bone formed as the bone-to-implant contact area at which evaluation is carried out includes the area over and above implant threads as well as the areas between threads. Only one study carried out elemental analysis (with the BIC I approach). Clearly all studies should include elemental analysis as it helps to assess the quality of BIC formed, information that is very useful when it comes to applying research outcomes to everyday clinical practice.
